# Sentiment Analysis of Texts on Public Health Emergencies Based on Social Media Data Mining

**DOI:** 10.1155/2022/3964473

**Published:** 2022-08-09

**Authors:** Nan Hu

**Affiliations:** School of Broadcast and Television, Communication University of China, Nanjing, China

## Abstract

**Background:**

Since the COVID-19 pandemic, social media has become an important arena for the public to transmit and exchange messages, feelings, opinions, and information about the epidemic. In the era of social media, many UGC contents from self-media and various information about the epidemic on social media have strong emotional colors. These contents are not only rich in resources for text sentiment analysis but also reveal the laws and characteristics of the evolution of users' emotional tendencies in public health emergencies. It even ties together the interaction between media content and society.

**Objective:**

As the Sina Weibo platform's characteristics of communication are real-time, open, and “many-to-many,” the objective of this study is to collect Weibo-blog contents tagged with the outbreak of COVID-19 in a certain metropolis in China and analyze the emotional evolution situation of Weibo-blogs of the unexpected public health emergency involved. This will provide a dynamic understanding of the mechanisms underlying the evolution of emotional conditions in the context of public health emergencies.

**Methods:**

This paper uses a Python crawler, the SnowNLP sentiment analysis model, and correlation analysis to calculate the emotional tendencies of the event “Covid-19 outbreak in a Chinese metropolis” on the Sina Weibo platform. The study was carried out in terms of the evolutionary stages of the event and the factors which induce it.

**Results:**

This paper revealed characteristics of time-varying laws and dynamic propagation of users' emotional evolution in public health emergencies. (1) This study refers to the life cycle model of COVID-19, combined with the statistics of the time series of the quantities of Weibo-blog posting, and divides the law of the quantities of Weibo-blog posting changing with the event into three stages: outbreak period, stalemate period, and resolution period. (2) Users' emotional tendencies are changeable and unstable which are easily induced by various factors. (3) There is a significant positive correlation between the reported confirmed cases and the quantities of Weibo-blog posts. (4) Individual emotional tendencies will have a positive changing trend with the public's average emotional tendencies after the event occurs. (5) There is no correlation between reposts, comments, and Weibo-blog emotional tendencies.

**Conclusion:**

The research found that, given staged evolution and repeated fluctuations of emotional tendencies, relevant departments should effectively use this law and set up different response plans according to different stages. In addition, what is highly coupled with users' emotional tendencies is not only the information about the virus but more large-scale infected by different intensities of emotions.

## 1. Introduction

Technological advancements in social media provide a faster, more accessible, and broader means of dissemination. The emotional interactions that users have when using these platforms will have a dynamic impact on their thoughts and actions, based on emotional responses to different information stimuli [1]. Specifically, during social media exposure, exposure to information shared by others can evoke different emotions such as indignation, joy, anger, or sadness due to the different personalities, tastes, and identities of users. Scholars such as Liu et al. [2] predicted users' emotional states (anxiety, frustration, anger, excitement, and confusion) on Weibo, compared the results with hot topics collected from social media, and found that there exists a significant correlation between them. As a result, the expression of public sentiment on online platforms can therefore be seen as a vane of real social trends. According to Bollen, public sentiment on the Internet can be influenced by economic, cultural, and political events in the real world, and conversely, it can have a series of “Butterfly effects” on the real world [3]. Other scholars have focused on the viral propagation of information and have arrived at contradicting conclusions from previous studies [4]. Although scholars have conducted rich and diverse research on text sentiment analysis based on different perspectives and methods, there are relatively few researches on sentiment analysis in thematic areas, especially in the context of a common topic facing the world today—the evolution of social media users' emotional in the context of public health emergencies. Second, although some scholars have sorted out and expounded on the evolution of the emotional tendencies of emergencies based on model construction and conducted empirical analysis through cases, however, it is limited to describing the process characteristics, and the analysis of the intrinsic patterns and triggering motives is not in-depth.

Text sentiment analysis is the process of analyzing, processing, summarizing, and speculating on subjective texts with emotional overtones, specifically by mining and analyzing the opinions, emotions, and polarities of texts through computational techniques and making categorical judgments on the emotional tendencies of texts. The original sentiment analysis originated from the analysis of words with emotional overtones [5]. For example, “friendly” is a positive word, while “unfriendly” is a derogatory word. With the emergence of a large number of subjective texts with emotional overtones on the Internet, researchers have gradually transitioned from the analysis of simple emotional words to complex emotional sentences. As a result, this paper assumes that “emotion” in text emotional analysis is a fairly broad concept, including the “emotion” commonly used to express love and hate (such as the abovementioned anxiety, frustration, or sadness), but also views in the text, that is, perceptions, ideas, and judgments. The research objective of the paper is to determine the sentiment tendency of the text, that is, whether the sentiment expressed by the user is positive or negative. This paper focuses on the evolution law and characteristics of users' emotional tendencies on social media platforms in the context of public health emergencies, not only the emotional tendencies are taken into account in the evolution model but also events, the quantities of newly confirmed cases, and the quantities of reposts, comments. The key elements are connected in series in the process of emotional tendencies evolution, in order to understand the internal mechanism of emotional tendencies evolution more deeply and dynamically under public health emergencies on the basis of integrating laws and motives. This paper takes Weibo's emotional tendency as the core to explore the following questions through the sentiment analysis of large quantities of Weibo-blogs.

Question 1: whether users' emotional tendencies are changing over time and showing a certain pattern?

Question 2: whether the quantities of Weibo-blog posted vary with the event and show a certain pattern?

Question 3: is there a correlation between the quantities of Weibo-blog posts and confirmed cases of COVID-19 on the same day?

Question 4: is there a correlation between the daily average emotional tendencies and the quantities of Weibo-blog posts with positive and negative emotional tendencies?

Question 5: how do Weibo-blog posts with different emotional tendencies relate to the quantities of reposts and comments?

## 2. Research Methods

### 2.1. Web Crawler

Sina Weibo is a social media platform that can publicly share and discuss individual opinions and activities. This paper uses Sina Weibo as a sampling pool and performs equal-proportion sampling based on the proportion of daily Weibo-blogs, so that the proportion of samples drawn daily is consistent with the quantities of total quantities of Weibo-blogs per day. The time period is selected from the municipal news release official account @Nanjing Announcement posted on the social media platform at 22 : 59 on July 20, 2021, “Notice of 9 positive cases of the Covid-19 at Nanjing Lukou International Airport” to August 9, 2021, “0 confirmed cases of the Covid-19.” After @Nanjing Announcement declared COVID-19 a pandemic, it was logical to assume that the general population started to be aware of the presence of the COVID-19 virus and be interested in symptoms and their health conditions. Also, they were exposed to the risk of the COVID-19 contraction before the government at all levels to do a good job strictly screening specific groups of people for possible infections. During this time period, ordinary people could discuss the COVID-19-related issues and share their personal experiences actively.

The Weibo-blogs which contain “Nanjing Epidemic” were crawled to obtain the following information: (1) username; (2) post time; (3) full texts; and (4) quantities of comments, reposts, and likes. Further, non-Unicode characters, missing, duplicate, and invalid posts are removed during the data cleaning process using the Pandas library. After cleaning, 15,100 valid posts will be further analyzed.

### 2.2. Machine Learning Methods

This paper uses SnowNLP, a third-party library for Python, to extract, analyze, and process emotional information (e.g., joy, frustration and anger) from Weibo texts. SnowNLP has many built-in functions such as sentiment analysis, text classification, and keyword extraction. In order to accurately measure the degree of emotionality, this study randomly selected 300 posts from the data set as training data and manually marked each post as positive or negative emotional, then inputs the updated emotional rating corpus file into SnowNLP for training and saving model, and then uses the Naive Bayes Theorem in the SnowNLP source code for sentiment analysis. Naive Bayes' Theorem can determine the emotional tendency of a reviewing text. The higher the degree of emotional tendency, the closer it is to positive emotion, otherwise, it is closer to negative [6, 7].

(1) $$\begin{array}{c} P\left(A\left|B\right.\right)=P\left(A\right)\frac{P\left(B\left|A\right.\right)}{P\left(B\right)}. \end{array}$$

The prior probability of the text *P*(pos) and *P*(neg) is calculated first, followed by the posterior probability *P*(word | neg) and *P*(word | pos). Finally, all texts were given an emotional tendency score on 0 to 1.

From the results of the prediction model calculation in Table 1, the research showed that the emotional tendency of the text “May Nanjing be safe” is 0.984, while the text that expresses fear and frustration, “How terrible! Why is it like that? ...”, the emotional tendency is 0.012, it can be seen that the analysis result of emotional orientation is consistent with cognition.

### 2.3. Related Analysis

Correlation analysis is an important means of determining the existence of associations between things, specifically by using data characteristics to verify the relationship between variables and the strength of the relationship.

## 3. Research Results

### 3.1. The Distribution Law of Emotional Tendencies

The linear fitting formula of splashed data is attitude = 0.404 − 0.002∗day, and the *R*-square value is 0.001.

Figure 1 shows the distribution of emotional tendencies of Weibo-blog over the whole period. The abscissa represents the quantities of days since the July 19 incident, and the ordinate represents the emotional tendency of Weibo-blog posts. It can be seen from the figure that the emotional tendency changes significantly with time variation, which indicates the characteristics of emotional changes on Weibo: people's emotional tendencies are affected by a variety of factors, and the emotional trends are fluctuating, unstable, and divergent. It is also obvious that in the early days of the incident, public opinions broke out in large quantities, and the emotional trend gradually declined. Negative emotions such as surprise and fear have been the dominant emotions on Weibo since the official announcement of the “9 Positive cases of Covid-19 at Nanjing Lukou International Airport.” Since the mainstream media began to guide public opinions, the overall emotion has stabilized, indicating that the media campaign has had a certain effect, but very negative emotions have always existed. In particular, negative emotions of various intensities were associated with specific events. For example, in the first nucleic acid test for the entire population, the anger was not only related to the shortage of medical and testing supplies, but also the home-stay order, quarantine measures, and the criteria for determining the yellow code. The above incidents caused Weibo users to question and express anger toward the government's antiepidemic work, and negative emotions broke out at this stage. In addition, the arrival of typhoon “fireworks,” the suspension of tourist attractions, and the strict management of transportation and epidemic control have further exacerbated fears. News such as “the neighboring district was building a square cabin hospital” and “47 new local confirmed cases in a single day” even made the fear of the public reach peak, and the emotional tendencies dropped to the lowest point 8-10 days after the outbreak of the incident. Afterward, news such as “Internet rumors of ‘red code' personnel buying medicines in pharmacies” were refuted, and the quantities of newly confirmed cases in a single day decreased day by day. The official announcement of “Nanjing Clearing” information was focused, and the overall emotional trend showed a positive trend.

### 3.2. Time Series Stage of the Quantities of Weibo-Blog Posts

Furthermore, this paper takes the life cycle model of COVID-19 as a reference [1], combined with the statistics of the time series of the quantities of Weibo-blog posts with event variation, and divides the law of the quantities of Weibo-blog posts with the event-variation into three stages (see Figure 2): outbreak period, stalemate period, and resolution period. During the outbreak period (1-6 days from the outbreak of the event), the quantities of Weibo-blog related to the event showed signs of rapid growth, with an average and median of about 853; during the stalemate period (7-15 days from the outbreak of the event), the quantities of Weibo-blog related to the incident fluctuated repeatedly, with an average and median of about 813; during the resolution period (16-21 days from the outbreak of the incident), the quantities of Weibo-blog related to the incident dropped significantly, with the average and median 513 or so.

### 3.3. The Correlation between the Quantities of Weibo-Blog Posts and New Confirmed Cases of COVID-19

By using the above table (see Table 2), the paper exams the correlation between the quantities of newly confirmed cases of COVID-19 and the quantities and expresses the relevant intensity with Pearson correlation coefficient. The correlation coefficient between confirmed cases of COVID-19 and the quantities is 0.507, which is significant at the 0.05 level. Therefore, it shows a significant positive correlation between the quantities of newly confirmed cases of COVID-19 and the quantities of Weibo-blog posts on that day.

### 3.4. The Correlation between the Daily Average Emotional Tendencies and the Quantities of Positive and Negative Emotional Tendencies on Weibo

As can be seen from Table 3, correlation analysis was used to study the correlation and intensity between the quantities of Weibo-blog with positive and negative emotional tendencies, the daily average emotional tendencies, and the quantities of days from the outbreak of the event. The specific analysis shows that the correlation coefficient between the quantities of Weibo-blog with positive emotional tendencies and the daily average emotional tendencies is 0.684, and the significance level is 0.01, indicating that there is a significant positive correlation between positive emotional tendencies and daily average emotional tendencies relation. The correlation coefficient between positive affective orientation and the quantities of days from the event was -0.604, and the significance level was 0.01, reflecting that there was a significant negative correlation between positive affective orientation and the quantities of days from the outbreak of the event. The correlation coefficient between the quantities of Weibo-blog with negative emotional tendencies and the daily average emotional tendencies was -0.764 and showed a significant level of 0.01, indicating that there was a significant negative correlation between negative emotional tendencies and daily average emotional tendencies. The correlation coefficient between negative affective tendency and the quantities of days from the outbreak of the event was -0.479 and reflected the significance at the 0.05 level, indicating that there was a moderate negative correlation between the negative affective tendency and the quantities of days from the outbreak of the event. This result shows that due to the existence of network empathy and herd mentality, individual emotional tendencies will have a positive changing trend with the public's average emotional tendencies after an event occurs.

### 3.5. The Relationship in Weibo with Different Emotional Tendencies and the Quantities of Comments and Reposts

It can be seen from Table 4 that correlation analysis is used to study the correlation and intensity between the number of reposts, comments, and likes, respectively, and the emotional tendencies of a single Weibo-blog. According to the results, it can be seen that there is no correlation between the number of reposts and the emotional tendency of Weibo-blog, the correlation coefficient value is 0.011, which is close to 0, and the *p* value is more than 0.05. Similarly, there is no significant relationship between the number of comments and the emotional tendency of Weibo-blog, and the correlation coefficient value is -0.001. No significant difference was found between the quantities of likes and the emotional tendency of Weibo-blog, and the correlation coefficient value was -0.007, indicating that there was no correlation between the likes and the emotional tendencies of Weibo-blog.

## 4. Discussions

### 4.1. “Burning Threshold,” “Emotional Slackness,” and “Public Opinion Rebound”

Based on the above study, we can see the segmented development of emotional tendency, which is that when online public opinion explodes under the stimulation of key events, emotional contagion drives online public opinion to reach the “burning threshold” quickly. The public opinion curve reaches a critical point when the public becomes “emotionally slack.” Since then, the attention rate has gradually cooled down. This is because there are a series of root causes for the change of online public opinion on emergencies, including changes in the event itself as well as changes in government behavior, users' interests, and media agendas. Online public opinion is a kind of “social consensus,” and as time goes by, without the intervention of new motivating factors, Internet users' emotions will gradually subside and develop in the direction of rationalization. From the perspective of the evolution of public opinion on the Internet in emergencies, the decay of public opinion is an inevitable phenomenon. At this stage, the public opinion entering the recession period will slowly subside and stabilize. However, due to the asymmetry of information, the extension of time and expansion of space, and the increase of public opinion elements, new focal issues arise again and the emotional tendency of netizens will fluctuate with the change of events, which also causes the rebound of public opinion heat. Given the segmental evolution and repeated fluctuations of emotional situations, relevant departments should effectively utilize this law and set up different response plans for different stages. For example, in the outbreak period, when the “burning threshold” is reached, the Weibo-blog with a high absolute value of emotional tendency is the densest. Therefore, paying attention to public opinion and accurately releasing authoritative news the first time is the priority. Relevant departments and relevant platforms can timely release relevant scientific information or conduct emotional guidance on social media platforms during this period. Another example is that relevant departments can unite with social media platforms and use artificial intelligence technology to regularly, repeatedly, and continuously release accurate and authoritative updates to the public and push emotional counseling information. This small-frequency, multidensity release rhythm is a powerful tool to effectively focus public opinion and attention.

### 4.2. “Infodemic”: The Dilemma of Emotional Susceptibility

Through the research on the correlation of Weibo-blog with different emotional tendencies and other related variables, it is found that what is highly coupled with the user's emotional tendencies is not only the information about the virus but also the large-scale infection of different intensity of emotions. The “Infodemic” is an increase in “susceptibility” to an infectious disease that infects our information culture [8]. One of the reasons is that we underestimated the amount of information flowing through social media. Social media in particular amplifies public emotions and disseminates this information to various nodes and spreads at an extremely fast speed [9]. Previous studies have shown that social media provides a source for the public in crisis to quickly find necessary information [10]. Unlike the spread of rumors in previous plagues, in today's social media era, everyone is a vocalist, and false information can spread across global social networks in just a day, spreading much faster than the development of the epidemic itself. The “Infodemic” is created and intertwined in the context of a real epidemic, thus making it more likely to lead to fear, stress, anxiety, and biased behavior, which is another cause of emotional susceptibility. Content-sensitive users, those who easily resonate with certain emotions, are more likely to overreact to relevant content. In the infodemic, content-sensitive users, users who easily empathize with certain emotions are more likely to overreact to related content. This has been observed in the bubonic plague in Chinatown communities and the Hantavirus infection in Michigan. For example, people are rude to those coughing in public places because they are afraid of being infected with the virus, which makes it easier for the specific emotional components transmitted by sensitive users to form a spiral. Moreover, the algorithm recommendation mode with traffic as the core further amplifies the effect of dramatic and conflicting information dissemination. Some of the self-media and marketing accounts publish a large number of intermingled emotional expressions, story narratives, and inflammatory contents, which are more likely to stimulate the sensitive nerves of the public and then trigger extreme emotions.

## 5. Conclusions

The research has found that, because of the staged evolution and repeated fluctuations of emotional tendencies, relevant departments should make effective use of this law and set up different response plans for different stages. In addition, it is not only information about the virus but also the mass contagion of different intensities of emotions that affect users' emotions. Finally, analyzing the evolution of emotional dynamics helps governments and authorities disseminate scientific outbreak data and verified news and provide timely guidance to counteract the emotional polarization caused by information asymmetry. There exist some shortcomings in this study. First, there is only one sample of public health emergencies, which cannot fully represent the characteristics of public health emergencies of the year, which may lead to certain differences in emotional and expression characteristics of Weibo-blog texts in the samples. Future research should seek to expand the type and quantities of events in the sample to capture public health emergencies in other areas, such as environmental protection and food safety. Second, the emotion categories were not subdivided in this study, and the classification of positive and negative emotions needs to be further optimized in future research.

## Figures and Tables

**Figure 1:** Splashed data graph of emotional tendencies with time-variation.

**Figure 2:** The time series of the quantities of Weibo-blog posts with event-variation.

**Table 1:** Naive Bayesian model prediction results.

Weibo text	Prediction results
#Nanjing epidemic #may Nanjing be safe.	0.983720876
Rainstorm in Henan, Nanjing epidemic, typhoon in Guangdong	0.983070539
#Rainstorm in Zhengzhou ## Nanjing epidemic# Hope everyone is safe and healthy!	0.999478028
#Nanjing epidemic #please be safe	0.918984165
#Nanjing epidemic# help, I just came back from a music festival, fortunately we are lazy, the day after the music festival is basically paralyzed in the hotel, but we went to the bar at night, ah ah ah ah ah ah, lack of money drove us not to fly, no tickets drove us to take a first-class seat, a lot less people, will not go out for two days, go for a nucleic acid test, so nervous!	0.0000000048
Severe flood disaster occurred in Zhengzhou, as well as Gongyi, Baoshui and other areas in Henan.# rainstorm in Henan# # 9 positive cases of COVID-19 detected at Nanjing Lukou International Airport##attention to COVID-19#severe flooding	0.527067843
#Rainstorm in Henan## Nanjing epidemic #play up, up, up! Hold on!	0.999947905
#Nanjing epidemic #oh my goodness!	0.64259687
#Rainstorm in Henan ##Nanjing Lukou epidemic # I am in Nanjing and my boyfriend is in Zhengzhou, hope it will not rain, hope everyone is safe & sound. Nanjing·Jianye Wanda Plaza	0.902680469
How scary the heavy rain in Henan is! Being trapped in the subway is the same as the scene in the movie. The epidemic situation in Yunnan is not good, and the epidemic situation in Nanjing is too difficult.	0.00050447
#Nanjing epidemic #no more!	0.755220441
The more I see the heavy rain in Henan and the epidemic in Nanjing, the more it really makes me sad. I can only pray for everyone's safe & sound!	0.065429261
#Nanjing epidemic # may Nanjing and Henan be safe & sound!	0.997548741
#Nanjing epidemic # the first piece of news is heavy rain in Henan, husband's elder sister is in Zhengzhou, at night, I was still worried about whether they would have something to eat, after playing with friends, my brother-in-law in Nanjing just said to watch the news when he got home. The second hot search is the Nanjing epidemic, oh, 9 cases! Nevertheless, I have a ticket back to Nanjing tomorrow, I have not seen my baby for days, I cannot change my ticket, be tangled be back or not, my mother said that you can touch on both sides.	0.000000010
#Nanjing epidemic # mask cannot be taken off!	0.424442214
#Nanjing epidemic # at this time, taking advantage of the chaos to slander the Chinese vaccine, suck the vaccine out of your body and get out of China like a toothpick, why is there always a group of people talking about Weibo when the country's in danger? Why are you a cool fish? It's disgusting enough, getting out of your foreign dad who likes you so much, China can go on without anyone.	0.0000021113
#Nanjing epidemic # I shivered in Jiangning. Nanjing·Wuyi Garden	0.008907375
I almost cried when watching the video and pictures of Zhengzhou Metro, too horrible! Life is too fragile & human beings are too tiny…Nanjing epidemic came with Zhengzhou flood, I cried, wanted to go back home, missing mum.	0.0000402421
#The rainfall within 3 days in Zhengzhou is as much as that of one year.#Nanjing epidemic # I took high-speed rail home from Nanjing yesterday, and still changing trains in Zhengzhou, really thrilling, hope everything is safe and sound!	0.064469709
#Nanjing epidemic #hold on, Nanjing!	0.628623876
#Nanjing epidemic # no matter how hot it is, you still have to wear a mask, OK?	0.092311253
#Nanjing epidemic #live in Jiangning, work in Jiangning, take shuttle every day at Nanjing South Metro Station with a huge flow of people, horrible! Horrible!	0.097829077
#Nanjing epidemic # get well soon	0.782278184
How terrible! Why is like that? Rainstorm in Henan & Nanjing epidemic very weak, life is too fragile.	0.012129899

**Table 2:** Correlation analysis between the quantities of Weibo-blog posts and the variables of newly confirmed COVID-19 cases.

	New confirmed cases of COVID-19
Quantities of Weibo-blog posts	0.507^∗^

^∗^ *p* < 0.05; ^∗∗^*p* < 0.01.

**Table 3:** Correlation analysis of the quantities of Weibo-blog posts with positive and negative emotional tendencies and the daily average emotional tendencies with time-variation.

	Quantities of positive emotional tendencies in Weibo-blog	Quantities of negative emotional tendencies in Weibo-blog
Daily average emotional tendencies in Weibo-blog	0.684^∗∗^	-0.764^∗∗^
Days from the outbreak of the event	-0.604^∗∗^	-0.479^∗^

^∗^ *p* < 0.05; ^∗∗^*p* < 0.01.

**Table 4:** Correlation analysis of Weibo-blog with different emotional tendencies and the quantities of comments and reposts.

	Quantities of reposts	Quantities of comments	Quantities of likes
Emotional tendencies of single post	0.011	-0.001	-0.007

^∗^ *p* < 0.05; ^∗∗^*p* < 0.01.

## Data Availability

The data that support the findings of this study are available from the corresponding author upon reasonable request.
